The article "A Feasibility Study on Smart Mattresses to Improve Sleep Quality" was published in 2021. Journal: J Healthc Eng.

# A Feasibility Study on Smart Mattresses to Improve Sleep Quality

**DOI:** 10.1155/2021/6127894

**Published:** 2021-08-03

**Authors:** Zicheng Zhang, Xinchen Jin, Zechuan Wan, Minghuan Zhu, Shanshan Wu

**Affiliations:** ^1^School of Information Management, Nanjing University, Nanjing, Jiangsu 210023, China; ^2^Advanced Medical Research Institute, Cheeloo College of Medicine, Shandong University, Jinan, Shandong 250012, China; ^3^School of Physics, Liaoning University, Liaoning, Shenyang 110036, China; ^4^Parmatech Medical Technologies Limited Company, Changzhou, Jiangsu 213000, China; ^5^Department of Endocrinology, Shandong Provincial Hospital, Cheeloo College of Medicine, Shandong University, Jinan, Shandong 250012, China

## Abstract

Good sleep quality is essential, especially for clinical users. Sleep disorders not only impair the success rate of treatment but also delay recovery. They can seriously interfere with treatment outcomes and even endanger a user's life. In this study, we created a smart mattress containing 10 × 18 air packs and control units. Each air pack contains a set of pressure and height sensors and two air valves. Each row control unit can detect and adjust the pressure and height of each air bag in the row. When the bed body is turned on, it automatically initializes, adjusts the state of each air bag to the same height and pressure, and enters a slow scanning state. When perceived objects or people are lying on the bed, the bed automatically perceives the human body structure and body pressure matrix, increases the scanning speed for more timely and accurate measurements of the digital matrix and forming pressure by matrix-normalized processing, and then uses local pressure variance detection to automatically adjust to the sleeping position of the human body and thus achieve a uniform force distribution and a comfortable state. Finally, pressure matrix binarization was used to match sleeping position templates to identify the best template for automatic recognition of the sleeping position. The experimental results show that the sleeping position recognition method has high accuracy, recall, and precision. Our mattress is designed with interfaces for external devices. In future research, the smart mattress can connect to an auxiliary part of a smart ecosystem consisting of a smart pill box, a smart lighting system, and a microclimate system, which is expected to yield a more comprehensive intelligent ward to explore the possibility of improving sleep quality.

## 1. Background

Most people work in the daytime and sleep at night; this rhythm of alternating sleep and wakefulness is known as the sleep-wake cycle [1]. Sleep is part of the sleep-wake cycle and is an autonomous, reversible behaviour controlled by an internal biological clock. Humans sleep for approximately one-third of their lives, which is a physiological process precisely controlled by several brain regions which is essential for healthy survival [2, 3]. Sleep is beneficial to the human body. Sleep allows the body to remove metabolic wastes produced by neurons in the brain and restores energy and strength, enhances immunity, promotes growth and development, improves learning and memory capacity, and contributes to emotional stability. Sleep is a necessary behaviour to maintain normal physiological activity [4].

In modern society, humans use artificial lighting. Competing pressures and bad habits continuously prolong our daily activity time, leading us to sleep too little and too poorly increasingly often. Such phenomena of abnormal sleep durations and abnormal behaviours during sleep are called sleep disorders [5]. According to a survey, nearly half of people have experienced sleep disturbances, potentially threatening their physical and mental health. Two-thirds of older adults and teenage students sleep less than eight hours [6–8]. Sleep disorders can also lead to asynchronous hormonal and metabolic regulation and metabolic abnormalities [9]. Users with chronic sleep disorders develop reduced glucose tolerance, hyperinsulinaemia, and insulin resistance, which can lead to cardiovascular disease [10] and diabetes mellitus in severe cases [11]. Sleep disorders affect the brain's neurons, leading to abnormal neurotransmitter secretion [12], disrupting cognitive function, and impairing learning and memory [13–17]. In addition, growing evidence shows that sleep disorders may lead to increased intrusive thoughts, affective disorder, and a higher risk of psychiatric disorders [18–20].

For clinical users, improving sleep quality is particularly important for the stability and improvement of their condition. Underlying diseases and noisy ward environments greatly compromise users' sleep quality, thereby impairing disease stability and recovery. Some users need hypnotics and psychological guidance to fall asleep during hospitalization. Therefore, how to improve sleep quality has become an urgent problem for clinical users and healthcare workers. Factors affecting sleep include physiological factors, psychological factors, and external environmental factors [21]. Optimizing external environmental factors such as temperature, humidity, light intensity, and atmospheric dust [22–24] is an effective means to improve sleep quality.

Comfortable bedding can create a more comfortable sleep environment. The breathability, insulation, elasticity, height, length, and even orientation of the bed should be in line with the human physiological structure. Developing a smart mattress that can optimize the external environment and be comfortable at the same time would be beneficial. Researchers have made many attempts to develop such a mattress. The gold standard of sleep monitoring is laboratory-based polysomnography [25]. Unfortunately, this method is expensive and inconvenient for users and researchers. Therefore, in recent years, many experts and scholars have started to use smart devices that can aid sleep to better monitor sleep and improve sleep quality. For example, commercially available smart bracelets can be used to monitor sleep based on actigraphy [26], but the data obtained are inadequate. An oximeter can monitor sleep based on blood oxygen and pulse [27] but cannot aid or improve sleep. Special mattresses can monitor sleep based on force sensors [28–30], but the existing mattresses are expensive and limited in function. Some researchers have invented devices that monitor sleep based on video and audio [31–33], but this kind of device is usually combined with other devices to function rather than working independently and has several privacy issues, rendering such devices unpopular. In addition, although some monitoring methods based on biological radar are accurate, they are expensive and difficult to promote [34–36]. Zhou Z et al. [37] proposed a single-layer, super soft intelligent textile, which can also be used for all-round physiological parameter monitoring and sleep healthcare. It can monitor dynamic changes in sleep posture, microbreathing, and Ballistocardiography (BCG). High sensitivity and good stability can facilitate sleep mattress use and increase the accuracy of sleep monitoring. In addition, intelligent textiles can be developed based on the human body and surrounding renewable energy, collect biological mechanical energy, human body heat energy, biological energy, solar energy, and hybrid forms of energy, be used to create intelligent equipment such as hand rings since electricity cannot be used for a long time and wearable electronic devices, and provide environmental protection energy [38]. Therefore, in follow-up research on intelligent sleep monitoring devices, more novel materials and auxiliary combinations of sleep monitoring devices should be considered.

In summary, as shown in Table 1, most monitoring devices detect physiological characteristics of the human body without initiating adjustments according to these characteristics. Little consideration has been afforded to whether and how pressure associated with the sleeping positions affects people's comfort during sleep. However, in this paper, a pressure sensor is used to monitor the sleep pressure of the human body and automatically adjust the pressure for an even distribution to try to make sleep more comfortable. This paper takes the intelligent mattress as the core and gives it good expansibility, supporting data access for external devices to facilitate their integration.

Our contributions are as follows: (1) We designed an intelligent mattress with the ability to recognize the pressure of the human body during sleep, which can recognize and image every part of the human body according to its structure. (2) We adopt a method based on local variance detection to automatically adjust the pressure on the body such that the pressure distribution during sleep is more uniform. (3) A sleeping position template is set up, and the human sleeping position is automatically recognized by analysing sampled data and matching the template.

## 2. System Design

The smart mattress has the functions of automatic recognition of body posture, automatic adjustment of hardness and height of relevant parts, autonomous learning, and smart detection and pushes. As regards recognition, the mattress can obtain users' sleep behaviour and sleep state data across the entire time domain and identify sleep-related data, as shown in Figure 1. As regards automatic adjustment, the mattress accurately detects changes in the body posture and the pressure distribution on the mattress while the user is asleep. In addition, according to its algorithm, it can apply real-time, independent smart adaptation/smart support for smoother and gentler dynamic mode adjustments. As shown in Figure 2, the mattress knows the user's sleep state and keeps the user comfortable and correctly balanced. When the user is awake, its main adjustment target is to keep the user comfortable; when the user is asleep, its main adjustment target is to keep the user in the right posture. As regards artificial smart recognition, this function is used to identify the most suitable sleep mode.

### 2.1. Design of the Smart Mattress

The main body of the mattress is composed of multiple air bags. The pressure borne by the air bag gives feedback to the smart adjustment system through the pressure sensor. Then, the smart adjustment system controls the air pump to inflate each air bag to adjust the hardness of the supporting point to provide a comfortable sleeping environment for the user. Users' heart rate and respiration can be detected, analysed, and recorded by measuring the frequency of vibrations of the air bag as part of the sleep quality analysis. Then, a series of sleep data can be used to provide better services for users such that the product can be individually tailored.

The air bag contains pressure and height detection sensors. The system automatically identifies the layout of the human body on the mattress according to the pressure distribution on the mattress and adjusts the air bag pressure at the corresponding position based on the distribution and the physiological structure of the human body. During adjustment, changes in pressure and height are fully considered.

#### 2.1.1. Data Monitoring Frequency Setting

At present, the data exist in 18 rows, which can monitor air bag height and pressure at different frequencies. The data are given by a host computer. In the event of power failure, the data are lost. We considered using an uninterruptible power supply to prevent data loss when the power is cut off. The required height and pressure of each air bag can be set independently. The pressure that each air bag can produce is the maximum pressure of the air pump. In the airtight state, the pressure borne by each air bag is greater than that of the air pump. A pressure-limit alarm is set, or the air outlet automatically opens to exhaust, to protect the air bag from damage. The pressure limit is saved by the single-chip microcomputer in each row. When the sleep mode is designed, the pressure of the air pump is taken as its implementable limit. The pressure of the air pump can be determined by the main control single-chip microcomputer and displayed instantly on the host computer. The height offset of each air bag is stored in the row-controlled single-chip microcomputer.

After powering on, the host computer can read in the stored height offsets, which are used to set the same corresponding height offset for each air bag when it is not loaded. The host computer can set and input the height offsets. After opening the exhaust valve, the pressure gradually stabilizes, and the stabilized pressure of each air bag is its pressure offset, which is processed in the same manner as the height offset. Each air bag can be set with an expected height and an expected pressure. Its control is limited by the pressure that the air pump can provide. When the pressure needs to be increased, a request can be sent to the host computer to turn on the air pump. To avoid competition with the I2C bus, how to merge into the message queue must be considered. The value (identity) of the air bag that needs to be operated can be evaluated first in the main control unit. If no current data are available, the detected information can be inserted into the message queue to obtain the detected data, and then the evaluation can be carried out. If the air pump is needed, it will be turned on. The number of air pumps that need to be turned on depends on the number of air bags that need to be operated. The air bags are evaluated and assigned to different levels. Then, according to the number of air bags at each level, the corresponding number of air pumps is turned on. To ensure that the air bag reaches the set value, the detection frequency of each air bag that needs to be operated is increased. After reaching the expected value, the detection frequency is set back to the initial value.

Regarding whether the heart rate and respiration need to be considered to process the data acquired at the increased frequency, we recommend that this is not necessary because normal air bag operation will be completed within a few seconds.

#### 2.1.2. Functions of the Host Computer

The pressure and height of each air bag are displayed. If a row is selected, the pressure and height of the current air bag will be displayed. If no such data are available, the fetching instructions can be sent directly. The expected pressure and height of each air bag can be set. An operation command can be input to open or close the valve of each air bag and transfer control to the test interface. In the test interface, the image display of the air bag is changed to scroll mode, and the statuses of a total of 20 air bag valves (each row) can be dynamically displayed. In the main interface, the pressure of the air pump output tube is increased instantaneously. The main interface has a mode control. For example, the added mode can be a control mode of a certain air bag point spreading to its surroundings. The mode can be set as an equation or a curve, and when a curve is chosen, a formula for the curve can be automatically generated as the mode acquired. An automatic analysis function is included. For areas with large data changes, the sampling frequency can be automatically increased to obtain heart rate and respiratory information. If no data change in the mattress occurs for a certain time, the judgement function determines whether this is because the user has left the mattress or because of an accident. A time setting function is also included. The automatic frequency reduction function and dehumidification function obtained by opening the air pump are active when the mattress is unoccupied.

A test program is used to perform the bundling operation of the airbag, including air intake and exhaust and reduction and shielding of the detected parameters, to fit the curves of the bundled area and to calculate differences between the measured and fitted parameters. The above tests are used to obtain the air bag layout and sensor layout to provide effective and executable solutions for productization. Due to the reduction in parameter information, a heat map will no longer be drawn. At this time, according to some parameters, an anthropomorphic pattern that is substantially similar to the user's body can be generated to facilitate user identification. If the lying posture needs to be judged, such as lying on the back and on the side, the sensor density in the local area should be noted. A schematic diagram of the control structure is shown in Figure 3.

#### 2.1.3. Control System Optimization

The reduction in the numbers of air bags and sensors can reduce the number of row control units. Reducing the number of sensors is more effective. At present, our detection unit has 10 channels (one for each row) of analogue-to-digital (AD) conversion; thus, each row control unit can control multiple rows of air bags. Because we use Serial Peripheral Interface (SPI) addressing, the number of valves is not restricted. At present, an 8-bit control method is adopted, which is synchronized with the 10-channel AD conversion and can still be set to 10 channels. The module under each air bag contains a sensor circuit and a valve control circuit. The valve control circuit is an addressing and latch circuit, and the sensor circuit is a gate circuit. We can try to integrate the two circuits into a chip to simplify the circuit form. The main control unit can greatly simplify the circuit by removing unnecessary precision clock circuits and retaining environmental monitoring circuits and communication circuits (universal asynchronous receiver-transmitter (UART) communication and Interintegrated Circuit (I2C) or controller area network (CAN) communication) to form the main control unit of a single bed. The main control unit is connected to an Android-based control system, which can be connected to two main control units to form the main control unit of a double bed. Control system add-ons include Bluetooth, Wi-Fi, ZigBee, USB outlets, and radiofrequency identification (RFID). Bluetooth is used to connect to the Android app. Wi-Fi is used to connect to the smart mattress control centre and the cloud (the smart device or app is not intended for transmitting large amounts of data but only for pushing processed information, program selection, related conclusive data, real-time data of certain physiological characteristics, etc.). ZigBee is used to connect to other smart devices, mainly including the ward environment maintenance system and smart bed lamps. Bluetooth can also connect to media players and other software. The environmental maintenance system includes the control of ward temperature. The software layer enhances the stability of the system and takes charge of restart functions after local problems, health diagnosis functions, and so forth.

#### 2.1.4. Air Pump Assembly Design

At present, although three air pumps are used, only one is used in the actual adjustment. After expansion of all air bags, using two is more than adequate, as they can already ensure a sufficiently fast response. The main work of this part is to reduce noise and simplify and facilitate the connections of pumps with the mattress. Sensors are added to facilitate the main control to detect the working efficiency of the air pumps (mainly the working pressure of the air pumps).

#### 2.1.5. Algorithm Design

Our design divides the bed body into 180 modules of 18 *∗* 10, and the size of each unit module is 10 cm *∗* 10 cm; thus, our intelligent mattress is 1.8 m *∗* 1 m in size. The value range of the pressure of the unit module is 0∼1,024. We divide the bed body according to the key structure of the human body, which mainly consists of the head, chest, waist, hips, and feet. When the user lies flat on the smart mattress, in terms of pressure distribution, the head and heel pressure is relatively large. Scanning from top to bottom in the pressure matrix, this unit module can be judged to have object pressure if it is greater than a certain threshold such that the user's general height can be measured. This paper establishes a general estimation of the user's height. When the number of unit modules increases, height recognition will be more accurate. The pseudocode of height recognition in this paper is as follows (see Algorithm 1).

After the head and feet of the human body are determined, several key parts of the human body can be determined from top to bottom according to the structure of the human body, including the chest, waist, hips, thighs, and calves. The segmentation method is shown in Table 2.

Because of the existence of a physiological curve, when the human body is in the supine position, the waist is in the vacated state. A waist in this state for a long time can cause the body to produce a tired feeling and affect sleep quality. When our mattress detects uneven stress at the waist position, it automatically injects gas into the uneven position to lift the air bag and average the pressure of the air bag such that the waist can be supported, therefore relieving fatigue. The variance in the pressure matrix is used as the evaluation function to assess the pressure of the air envelope. Smaller variance in the pressure matrix value of the force surface corresponds to more uniform force and greater comfort. The pseudocode for automatic adjustment is as follows (see Algorithm 2).

After obtaining the pressure matrix of the human body, we must recognize the sleeping position of the human body, which can be modelled as the classification of the pressure matrix. In fact, the classification of the pressure matrix is very similar to the image classification, both of which are matrix classifications. Therefore, we introduce the classification method in image processing in this paper for recognition of the sleeping position. First, we define four sleeping positions as follows: kneeling position, supine position, prone position, and lateral position. Of course, as the number of users slowly increases, the number of postures also increases. Due to the limited labelling data, the template-based sleeping position recognition method was adopted in this study. The specific methods are as follows. First, grey processing was performed on the pressure matrix PM, and the pressure value was processed to between 0 and 255 according to the following formula:

(1) $$\begin{array}{c} pm\left[i,j\right]=\text{round}\left(\frac{pm\left[i,j\right]}{\max\left(pm\right)}\right)\times 255,\;\;i\in \left[1,\ldots ,18\right],j\in \left[1,\ldots ,10\right], \end{array}$$

where round represents the rounding function and max represents the maximizing function.

After processing, the pressure matrix was binarized according to formula (2) to highlight the contour.

(2) $$\begin{array}{c} pm\left[i,j\right]=\left\{\begin{array}{cc} 255, & \text{if }pm\left[i,j\right]>\varepsilon \;i\in \left[1,\ldots ,18\right],j\in \left[1,\ldots ,10\right],\\ 0, & \text{else.} \end{array}\right. \end{array}$$

Matrix V is obtained by the “and” operation between the pretreated pressure matrix U to be identified and the sleeping position matrix T in the sleeping position template library. The common part obtained and the matrix of the sleeping position to be recognized are logically “XOR” operations, and the excess part of the matrix of the sleeping position to be recognized is matrix X. After logical XOR operation between the obtained common part and the template sleeping position matrix, the redundant part of the template sleeping position matrix W is obtained. We define *T* as the number of values in matrix *M* of each template sleeping position matrix, *U* as the number of values in the pressure matrix to be recognized, and *V* as the number of values in matrix V of the common parts of matrix U and matrix T, 255. Matrix W defines *W* as a number of values of 255, *X* is defined as a number of values of 255 in matrix X, and the expression of the discriminant function is constructed as shown in the following formula:

(3) $$\begin{array}{c} Y_{i}=\frac{V_{i}}{W_{i}/T\times X_{i}/U\times \sqrt{{\left(T_{i}-TUV_{i}\right)}^{2}+{\left(U-TUV_{i}\right)}^{2}+{\left(V_{i}-TUV_{i}\right)}^{2}/2}}, \end{array}$$

where *TUV*=(*T*+*U*+*V*)/3,*i* is the serial number of the template library, and the sleeping position template *i* corresponds to the maximum similarity coefficient max(*Y*_*i*_) for identification of the sleeping position. The identification process is shown in Figure 4.

## 3. Experimental Results

### 3.1. Setting of Experimental Parameters

In Table 3, *δ* is the pressure threshold for pressure determination, *γ* is the variance threshold for automatic adjustment, and *ε* is the pressure threshold for binarization.

### 3.2. Experimental Study

Table 4 describes the detailed information of the 5 subjects, including age, sex, height, and weight.

The experimental results are shown in Table 5: accuracy, recall, precision, and F1_score.

Figure 5 is the confusion matrix of the experimental results. According to the experimental results, recognition of the kneeling position, supine position, and prone position is more accurate. Identification of the lateral position in people with low body weights (52 kg and 55 kg) will produce errors because the lateral lying position is very similar to the supine position. When the lateral lying position is straight without an obvious arch and the body is light, the distribution of hands cannot be distinguished, resulting in an inability to clearly distinguish the supine and lateral lying postures. A lighter body is more difficult to detect, which is especially true when a person sleeps or lies on their side and remains straight with the hands drawn towards the body; at this point, the supine position and the side position occupy the same amount of air sac, complicating differentiation. In contrast, when the body is heavier, the contrast is more obvious, and the distinction is much easier. Of course, in the lateral decubitus position, the arched arrangement can also be accurately identified.

We have completed research and development of the first-generation smart mattress, as shown in Figure 6.

The first-generation smart mattress can already recognize the posture of the human body. As shown in Figure 7, it can correctly recognize the posture of the human body and the pressure exerted by the body on the mattress. A darker colour in the figure corresponds to greater pressure on that part of the mattress.

When the smart mattress detects uneven stress on the human body, the air pump will be turned on, and the stress on the user during sleep will reach a uniform distribution through smart adjustment, thus improving the user's sleep quality. The effect is shown in Figure 8.

## 4. Conclusion and Discussion

This article discusses the function, structure, and design method of the mattress. The innovative smart mattress controls its air bags to adjust the support points of the mattress through embedded technology. With this study, we completed research and development of first-generation products and achieved satisfactory testing results. A comparison between our mattress and a Sleep Number mattress is shown in Table 6. Overall, compared with the Sleep Number mattress, the mattress designed in this study is not only a mattress but also a system—a smart mattress that can be embedded with AI to achieve adaptive adjustment.

## 5. Limitations and Solutions

### 5.1. Limitations

1. The valves that control inflation and deflation of the bag are not integrated, resulting in a large number of valves
2. The height of the air pocket is low, the deformation space is small, and more modes cannot be formed
3. The air bag layout and the support structure of the mattress are relatively rigid, and the soft structure and rigid structure of the bed body cannot adapt to each other
4. With less test data, the sleeping position recognition method based on template matching was adopted

### 5.2. Solutions

1. Integrate the inflating and deflating valves of the bag to reduce the number of valves
2. Increase the height of the air bag such that its deformation space is larger, which is convenient for incorporating more postures
3. To improve the layout of the air bag and the support structure of the mattress, the support structure can drive the air bag to deform together; that is, the soft structure of the bed body and the rigid structure can adapt to each other such that the mattress can tilt and adapt to the sitting posture
4. By increasing the test data and using the machine learning method to annotate a large amount of sleeping position data, the recognition accuracy can be further improved

## 6. Future Prospects

In the future, a smart ward will be equipped with a microclimate system to regulate the temperature, humidity, and atmospheric dust in the ward. A smart lighting adjustment system provides a warm visual atmosphere for users, and a health and sleep emergency system provides health monitoring of the user. The composition of a smart ward is shown in Figure 9. We also designed a sleep emergency smart pill box to provide a safety measure for users with acute diseases. Once any abnormality in the body or abnormal data are detected, this information will be sent to a data centre, a nurse station, and a resident doctor simultaneously. At the same time, the smart pill box will match life-saving drugs to the user's symptoms. The composition of the sleep emergency smart pill box is shown in Figure 10.

## Figures and Tables

**Figure 1:** The process of automatically recognizing sleeping position. *Note*. The sleeping position in this figure includes lying supine, lying on the left, lying on the right, and lying prostrate.

**Figure 2:** The process of automatic correction of body posture during sleep. *Note*. This figure depicts that the force becomes uniform after adjustment from the uneven force.

**Figure 3:** Schematic diagram of the control structure. *Note*. This figure describes the hardware working principle and composition of the smart mattress.

**Figure 4:** The process of sleeping position recognition.

**Figure 5:** Confusion matrix of four kinds of sleeping position recognition results.

**Figure 6:** Physical map of smart mattress.

**Figure 7:** Four kinds of human sleeping position recognition. (a) Kneeling position. (b) Supine position. (c) Prone position. (d) Kneeling with ground support.

**Figure 8:** The comparison of automatic adjustment of the smart mattress. (a) Nonuniform pressure distribution. (b) Uniform pressure distribution.

**Figure 9:** Diagram of the smart ward's composition. *Note.* The concept of smart ward is composed of smart lighting and entertainment, air and temperature, and health monitoring.

**Figure 10:** Diagram of the medical and health platform. *Note.* The concept of smart ward is composed of smart housekeeper, data integrated monitoring headrest, and sleep emergency smart pill box.

**Algorithm 1:** Height recognition pseudocode.

**Algorithm 2:** Automatic adjustment pseudocode.

**Table 1:** Comparison of the different aspects by smart devices.

Sleep monitoring method	Sensor	Monitored data	Test parameters	Advantages	Disadvantages
PSG	Electrode	Human electrical signal	Electroencephalogram, eye movement, mandibular electromyogram, electrocardiogram, oral and nasal airflow, chest and abdominal movements, snoring, blood oxygen saturation, blood pressure before and after sleep	A variety of physiological indicators can be monitored to identify sleep stages	Complicated operation, which affects subjects' sleep quality, and the cost of sleep assessment is high

Oximetry	Pulse oximeter	Changes in blood volume in the human arteriolar bed	Pulse rate, blood oxygen saturation, perfusion index	The disturbance is small, and simple sleep staging can be realized	Mainly used in laboratory research and difficult to use at home

Intelligent bracelet	Body motion recorder	Movement of the human body in the *X*-, *Y*-, and *Z*-axes	The occurrence and degree of body motion signals, body motion amplitude, and body motion frequency	Low cost, low interference, continuous monitoring for a long time	Too little data are collected to achieve sleep staging

Sleep mattress	Force-sensitive transducer	Pressure change signal between the user and the mattress	Respiratory rate, body movement	Both comfort and the monitoring function allow sleep staging	Difficult to carry and expensive

Video and audio	Infrared, sound sensors	Changes in movement and nasal and mouth sounds during sleep	The state of sleep and wakefulness	The disturbance is small, and simple sleep staging can be realized	Privacy issues

Biological radar	Biological radar	Body movement signal, respiratory signal	Respiratory rate, body movement	Without interference, various physiological parameters can be monitored at the same time to realize sleep staging	Expensive and difficult to promote

Comparing various smart devices commonly available on the market in terms of sensors, monitored data, test parameters, advantages, and disadvantages.

**Table 2:** Body parts and corresponding mattress positions.

Body parts	Mattress line number
Head	1∼2
Shoulder to the chest	3∼6
Waist	7∼8
Hips	9∼10
Thighs	11∼13
Calves	14∼16

**Table 3:** Experimental parameters settings.

Parameter	Value	Note
*δ*	1020	Pressure threshold
*γ*	3	Variance threshold
*ε*	150	Binarization threshold

**Table 4:** Data of the experimenters.

Number	Age	Sex	Height	Weight
1	25	Female	1.65	55
2	35	Male	1.72	70
3	42	Male	1.75	67
4	55	Female	1.55	60
5	40	Female	1.62	52

**Table 5:** Experimental results.

Indicators	Value
Accuracy	0.900
Recall	0.900
Precision	0.929
F1_score	0.896

**Table 6:** Function comparison between our product and the Sleep Number mattress.

Function	Our product	Sleep Number
Body posture recognition	Yes	No
Automatic adjustment	180 airbags	Single airbag

## Data Availability

No data, models, or codes were generated or used during the study.
